# Using Haemocoagulase Agkistrodon in Patients Undergoing Transurethral Plasmakinetic Resection of the Prostate: A Pilot, Real-World, and Propensity Score-Matched Study

**DOI:** 10.1155/2022/9200854

**Published:** 2022-06-22

**Authors:** Cong Zhu, Lan Yang, Hao Zi, Bing-Hui Li, Qiao Huang, Meng-Xin Lu, Xiao-Dong Li, Xuan-Yi Ren, Hua Tao, Hankun Hu, Xian-Tao Zeng

**Affiliations:** ^1^Department of Urology, Zhongnan Hospital of Wuhan University, Wuhan 430071, China; ^2^Center for Evidence-Based and Translational Medicine, Zhongnan Hospital of Wuhan University, Wuhan 430071, China; ^3^Division of Medical Affairs, Zhongnan Hospital of Wuhan University, Wuhan 430071, China; ^4^Department of Urology, Huaihe Hospital of Henan University, Kaifeng 475000, China; ^5^Department of Urology, Kaifeng Central Hospital, Kaifeng 475000, China; ^6^Department of Pharmacy, Zhengzhou Second Hospital, Zhengzhou 450006, China; ^7^Department of Pharmacy, Zhongnan Hospital of Wuhan University, Wuhan 430071, China

## Abstract

**Objectives:**

To compare the clinical outcomes of using different hemostatic agents after transurethral plasmakinetic resection of the prostate (TUPKP) in benign prostatic hyperplasia (BPH) patients.

**Methods:**

The patients were divided into 5 groups according to the hemostatic agents used after TUPKP, including the haemocoagulase agkistrodon for injection (HCA), hemocoagulase for injection (HC), hemocoagulase bothrops atrox for injection (HCB), ethylenediamine diaceturate injection (EDD), and tranexamic acid (TXA). Propensity score matching was performed based on age, body mass index, prostate volume, hypertension status, fasting blood glucose, smoking, and drinking history. The hospitalization time, bladder irrigation time, indwelling catheterization time, the patency of urine flow, and blood transfusion records were used as outcome indicators to compare the clinical effects of these five agents.

**Results:**

We finally matched 65 pairs receiving HCA or HC, 71 pairs receiving HCA or HCB, 38 pairs receiving HCA or TXA, and 29 pairs receiving HCA or EDD. Compared with HC, HCA given during the perioperative period significantly reduced the median hospitalization time [7.00 days (5.00, 8.00) vs. 9.00 days (8.00, 10.00); *p* < 0.001] and median catheterization time (109.00 hours [88.00, 129.00] vs. 164.00 hours [114.00, 189.00], *p* < 0.001). Compared with EDD, the median hospitalization time (7.00 days [6.00, 8.00] vs. 10.00 days [8.00, 11.00]; *p* < 0.001) and median catheterization time (113.00 hours [95.00, 143.00] vs. 160.00 hours [139.00, 168.00]; *p* < 0.001) were also significant shorter in HCA group. Compared with HCB, median bladder irrigation time (45.00 hours [27.00, 71.00] vs. 49.00 hours [45.00, 72.00]; *p* = 0.04) was shorter in the HCA group. However, there were no statistical differences in outcomes between HCA and TXA.

**Conclusions:**

HCA probably has an advantage over HC, HCB, and EDD in reducing the hospitalization time, catheterization time, and bladder irrigation time among BPH patients undergoing TUPKP.

## 1. Introduction

Benign prostatic hyperplasia (BPH) is a common urinary system disease in elderly men, often leading to lower urinary tract symptoms (LUTS), which seriously affect the patients' quality of life. In 2019, it was estimated that the incidence of BPH was as high as 2298.45/100,000 in the age group of 65-70 years [1]. The burden of BPH will further increase as global population ageing accelerates [2]. When conservative and pharmacological treatments are not effective, surgery is often unavoidable. Transurethral resection of the prostate (TURP) is the preferred surgical paradigm for the treatment of BPH. However, traditional monopolar TURP has two main limitations [3, 4], one is water toxicity which can lead to negative outcomes and the other is poor hemostasis. In 2011, the European Association of Urology included transurethral plasmakinetic resection of the prostate (TUPKP) in its guidelines and recommended it for the first time, because of the benefits of less intraoperative bleeding and fluid absorption and fewer postoperative complications [5–7]. Even though various devices and techniques have been developed, perioperative bleeding is still a challenge for urologists, given that it may lead to prolonged bladder irrigation time and hospitalization time [8].

The use of hemocoagulase, tranexamic acid, and ethylenediamine diaceturate in hemostasis in TURP patients have been reported in previous studies [9–11]. However, there were few studies comparing the clinical prognostic effects among these different hemostatic agents on patients undergoing TUPKP. Haemocoagulase agkistrodon for injection (HCA) is a national first-class drug in China with a good hemostatic efficiency and is safe when used in capillary bleeding from abdominal incisions having few side effects [12, 13]. Therefore, we compared the clinical prognostic effects of HAC with other hemocoagulase drugs, tranexamic acid (TXA), and ethylenediamine diaceturate (EDD) on patients undergoing TUPKP.

## 2. Methods

### 2.1. Study Design and Subjects

This was a preliminary, multicenter, real-world, and propensity score-matched study. The subjects were selected from a prospective study, the Bladder Cancer and Benign Prostatic Hyperplasia Study in Chinese Populations, which ran from September 2016 to November 2018 [10, 14–19]. This study was reviewed and approved by the Committee for Ethical Affairs of the Zhongnan Hospital of Wuhan University. All participants signed written informed consent before enrollment.

Patients with confirmed BPH who had undergone TUPKP were included, while patients with urinary malignancies, urinary tract infections, and abnormal coagulation disorders were excluded. The included patients were divided into five groups according to the real-world data of hemostatic agents: HCA (brand name: Suling), hemocoagulase for injection (HC, brand name: Bangting), hemocoagulase bothrops atrox for injection (HCB, brand name: Baquting), TXA, and EDD; all of them were intravenously administered after TUPKP. Each patient may have been given more than one coagulant. When comparing two specific hemostatic agents, patients who had been given only one specific hemostatic agent were included in treatment groups.

### 2.2. Measurements and Data

Detailed demographic characteristics and medical history were collected, including age (years), body mass index (BMI, kg/m^2^), hypertension status, smoking, and drinking history. Physical examination data were recorded, including prostate volume (PV, mL), systolic pressure (SBP, mmHg), diastolic pressure (DBP, mmHg), and fasting blood glucose (FBG, ng/mL). These data served as baseline characteristics of each enrolled patient. Moreover, details of hemostatic agents received by each patient after operation were recorded. The hospitalization time (days), bladder irrigation time (hours), catheterization time (hours), patency of urine flow, and blood transfusion records served as outcome indicators to compare the clinical effects of these hemostatic agents.

BMI (kg/m^2^) was calculated by dividing weight in kilograms by the square of height in meters. SBP and DBP were measured according the standard method recommended by the American Heart Association guidelines [20]. Prostate ultrasound was used to measure the largest anteroposterior height (*H*, cm), transverse width (*W*, cm), and cephalocaudal length (*L*, cm) of prostate, and prostate volume (mL) was calculated using the ellipsoid formula [21] *PV* = (*π*/6) × *H* × *W* × *L*.

### 2.3. Statistical Analysis

Propensity score matching (PSM) was used to reduce the bias and imbalance of confounding variables that is present in observational studies [22]. In this study, age, BMI, PV, hypertension status, FBG, and history of smoking and drinking were used to estimate the propensity score. A 1 : 1 greedy match was performed base on a caliper width of 0.2 for the propensity score. Categorical variables were expressed as frequencies (percentage), and continuous variables were described using mean ± standard deviation or median (the first quantile, the third quantile) based on normality test. Before and after PSM, patients' characteristics and outcomes were compared between HCA and the other four groups, using chi-squared tests for categorical variables and Student's *t*-test (or Wilcoxon rank-sum test) for continuous variables, as appropriate. All analyses were carried out using the SAS software, version 9.4 TS1M6 (SAS Institute Inc., Cary, NC).

## 3. Results

### 3.1. Patients' Characteristics before PSM

Overall, 113 patients received HCA after TUPKP, while 86 patients received HC, 99 patients received HCB, 49 patients received TXA, and 37 patients received EDD. Compared with patients who received only HCA or HC, the median age of the two groups were 73 (66.00, 79.00) and 71 (66.00, 76.00) years old (*p* = 0.14), respectively. The median BMI of two groups were 23.36 (20.62, 25.53) kg/m^2^ and 23.05 (20.76, 24.57) kg/m^2^ (*p* = 0.49), the mean prostate volume were 51.65 mL (32.46, 81.68) and 50.31 (38.73, 71.42) for the two groups (*p* = 0.96). Likewise, there were no statistically significant differences between the two groups in the SBP, DBP, FBG, hypertension status, and history of smoking and drinking (all *p* > 0.05) (Table 1).

There were no significant statistical differences in baseline characteristics between the patients receiving HCA and those receiving HCB. There were no differences in baseline characteristics between patients receiving HCA and patients receiving TXA (Tables 2 and 3). However, the SBP was significantly higher (*p* = 0.4) in patients who had received HCA (132.00 mmHg [121.00, 142.00]) than in patients who had received EDD (126.00 mmHg [116.00, 130.00]). In addition, the proportion of patients with smoking history in the EDD group was higher than that in the HCA group (56.76% vs. 25.66%) (*p* < 0.001) (Table 4).

### 3.2. Patients' Characteristics after PSM

After PSM, we matched 65 pairs who had received HCA or HC, 71 pairs received HCA or HCB, 38 pairs received HCA or TXA, and 29 pairs received HCA or EDD according to the propensity score. Overall, there was no significant statistical difference in the baseline characteristics of the four matched treatment groups (all *p* > 0.05) (Tables 1–4).

### 3.3. Outcome Difference of Each Matching Group

The median time of hospitalization of the HCA group was 7.00 days (5.00, 8.00), which was significantly shorter than the 9.00 days (8.00, 10.00) of the HC group (*p* < 0.001). The median catheterization time was also shorter in the HCA group (109.00 hours [88.00, 129.00]) than in the HC group (164.00 hours [114.00, 189.00]) (*p* < 0.001). Nevertheless, the median bladder irrigation time (*p* = 0.06), patency of urine flow (*p* = 0.68), and blood transfusion records (*p* = 1.000) showed no statistical differences between the two groups. The median hospitalization time (7.00 days [6.00, 8.00] vs. 8.00 days [7.00, 10.00]) (*p* < 0.001), median bladder irrigation time (45.00 hours [27.00, 71.00] vs. 49.00 hours [45.00, 72.00]) (*p* = 0.04), and median catheterization time (114.00 hours [88.00, 143.00] vs. 141.00 hours [120.00, 166.00]) (*p* < 0.001) were significantly shorter in the HCA group compared with the HCB group (Table 5).

No significant difference was recorded when comparing the outcome indicators of patients receiving HCA and patients receiving TXA (all *p* > 0.05). The median hospitalization time (7.00 days [6.00, 8.00] vs. 10.00 days [8.00, 11.00]) (*p* < 0.001) and median catheterization time (113.00 hours [95.00, 143.00] vs. 160.00 hours [139.00, 168.00]) (*p* < 0.001) of patients who had received HCA were significantly shorter than that of patients who had received EDD. The median bladder irrigation time, patency of urine flow, and blood transfusion records showed no significant differences between the two groups (*p* > 0.05) (Table 6).

## 4. Discussion

In this propensity score matching study, we compared the clinical effects of HCA with 4 clinically commonly used hemostatic agents in BPH patients receiving TUPKP. Overall, the use of HCA for patients during the perioperative period significantly reduced the hospitalization time and catheterization time compared with HC and EDD. Bladder irrigation time was also shortened when compared with HCB. However, there were no statistical difference in all outcome indicators between HCA and TXA. Our results suggest that postoperative use of HCA and TAX in patients with BPH undergoing TUPKP can effectively reduce the patient and medical burden compared with HC, HCB, and EDD.

TUPKP has advantages in reducing TURP syndrome, clot retention, irrigation, and catheterization duration [23]. Nonetheless, perioperative bleeding management remains a priority for BPH patients [8], for which increases the operation time, irrigation fluids, the risk of TURP syndrome and sepsis, hospitalization time, catheter obstruction, and transfusion [8]. Our results indicated that BPH patients using HCA had the significantly shorter hospitalization time than those using HC, HCB, and EDD. Reducing hospitalization time means reducing the financial burden and improving patient comfort, as well as facilitating the efficient use of medical resources [24]. Previous clinical research found that HCB can significantly shorten the hospitalization time and prothrombin time among BPH patients undergoing TUPKP, but this study did not compare HCB with other hemostatic agents [10]. These results affirm the positive effect of hemocoagulase in BPH patients receiving TUPKP; however, HCA significantly shortened the hospitalization time of patients compared with HCB. We speculate that it may be related to the single component, high purity, and high active potency of HCA, which can significantly reduce the bleeding time and volume without causing thrombosis [25–27].

We further compared the bladder irrigation time and catheterization time among BPH patients using different hemostatic agents after TUPKP. We found that HCA significantly shortened bladder irrigation time and catheterization time than HC, HCB, and EDD, suggesting better hemostasis effect. Although studies of HCA in patients with TUPKP are lacking, phase II and III clinical trials of HCA have demonstrated its effectiveness in reducing hemostatic time, bleeding volume, and bleeding volume per unit area during abdominal surgery [26, 28]. Perioperative intravenous HCA was also found to significantly reduce blood loss and blood transfusion in elderly fracture-related hip arthroplasty without increasing short-term adverse event rates and increase postoperative subacute hemoglobin and coagulation factor levels [29]. This also demonstrates the safety of HCA in the elderly, since patients with BPH requiring surgical treatment are generally elderly.

The antifibrinolytics TXA was also used to reduce perioperative bleeding in TURP patients [30, 31]. In our study, HCA and TXA showed no significant differences in postoperative indicators of concern. A meta-analysis indicated that TXA effectively reduced perioperative blood loss compared with placebo in patients undergoing TURP; however, there was no significant improvement in preventing transfusions and increasing hemoglobin [32]. The hemostatic effects of EDD and TXA have been compared, and EDD was found to be more effective than TXA in reducing blood loss in open prostatectomy patients [11]. Our results showed that HCA was more effective than EDD in reducing the hospitalization time and catheterization time among patients undergoing TUPKP, which may suggest that HCA is more suitable for minimally invasive surgery than EDD. It is known that prostate tissue contains a large amount of tissue plasminogen activator, and urine flow contains high concentrations of urokinase, which are released in large quantities during prostatectomy to activate the fibrinolytic system [33, 34]. The HCA can antagonize this effect by promoting the synthesis of fibrin, and TXA reduces the degradation of fibrin by inhibiting the binding of fibrinolytic enzyme to fibrin. However, EDD inhibits the fibrinolytic system by inhibiting the synthesis of fibrinolytic enzyme, it does not directly protect fibrin from degradation or promote fibrin aggregation as the two former drugs do. Therefore, we inferred that this may be the reason that why HCA and TXA were more effective in reducing hospitalization time and catheterization time than EDD in patients after TUPKP.

In addition, some urologists selectively use 5*α*-reductase inhibitors (5-ARIs) before surgery to reduce intraoperative and postoperative bleeding in patients with large prostate volumes, hematuria, or high risk of bleeding [35]. Some studies showed that 5-ARIs can reduce blood loss or transfusion requirements in BPH patients undergoing TURP [36–38]. However, other studies did not find significant differences between 5-ARIs and placebo in blood loss during surgery, excessive or severe bleeding, or retention of clots [39, 40]. No studies compared the role of 5-ARIs and HCA in perioperative prophylaxis or hemostasis in patients with BPH, but the different mechanisms and ways of use determine the scope of their use. Compared with HCA, 5-ARIs reduces prostate blood flow by downregulating vascular endothelial growth factor, which is typically administered before surgery for 2-4 weeks [37, 38]. On the other hand, side effects of 5-ARIs should also be considered such as hypaphrodisia, erectile dysfunction, ejaculatory dysfunction, and potential depression [41].

Although the efficacy of the hemostatic agents mentioned above has been proved in related studies, their safety is still a concern of urologists. Several studies have reported that HCA did not show significant complications [25, 28, 29, 42, 43]. Moreover, it was reported that 36% to 44% of patients undergoing TURP used anticoagulant or antiplatelet drugs [44]. Although the safety of TUPKP for patients receiving anticoagulant and antiplatelet drugs has been explored, there is still an increased risk of perioperative bleeding among these patients [45, 46]. A study found that HCA exerted hemostatic effect without causing thrombosis [25]; however, more clinical trials are still needed to support the safety and effectiveness of perioperative use of hemocoagulase in TUPKP patients needing oral anticoagulant drugs or antiplatelet drugs. Recent studies have shown that topical administration of hemocoagulase was effective in reducing bleeding, pain, and swelling after tooth extraction and accelerating the wound healing process [47, 48]. Obviously, the drug potential of hemocoagulase remains to be developed, and its application prospect in urology still needs more exploration. Overall, we still need to pay attention to the scope of application of hemocoagulases, monitor the coagulation function of patients, and adjust the dosage according to the specific conditions of patients.

Our research also had some limitations. Firstly, we chose the hospitalization time, catheterization time, and bladder perfusion time as outcome variables rather than the more intuitive indicators of hemostatic effect, such as volume of blood loss and hemoglobin reduction ratio, because we considered the heterogeneity between patients and the influence of confounding factors. Hospitalization time and catheterization time are also more in line with the current concept of enhanced recovery after surgery. Moreover, administration period of hemostatic agents is a factor needed to be taken into account in future studies. Second, propensity matching was used to make baseline characteristics more balanced between treatment groups, but it also reduced the sample size of each group. Thirdly, due to the limitation of the available data, the study did not compare the health economics outcomes of these drugs. In addition, this study was only based on the Chinese population, and its universality needs to be verified in other regions of the world.

## 5. Conclusion

In conclusion, our results indicated that HCA had an advantage over other types of hemocoagulase and EDD in reducing the hospitalization time, catheterization time, and bladder irrigation time among BPH patients undergoing TUPKP, but such differences were not found between the HCA and TXA. We also recommend performing more randomized controlled trials with large sample sizes to confirm these results.

## Figures and Tables

**Table 1:** Baseline characteristics of patients used haemocoagulase agkistrodon for injection or hemocoagulase for injection before and after propensity score matching.

Baseline	Before propensity score matching			After propensity score matching		
	Haemocoagulase agkistrodon (*N* = 111)	Hemocoagulase (*N* = 86)	*p*	Haemocoagulase agkistrodon (*N* = 65)	Hemocoagulase (*N* = 65)	*p*
Age (years)	73.00 (66.00, 79.00)	71.00 (66.00, 76.00)	0.14	70.00 (65.00, 77.00)	69.00 (66.00, 76.00)	0.86
Body mass index (kg/m^2^)	23.36 (20.62, 25.53)	23.05 (20.76, 24.57)	0.49	23.42 ± 3.82	23.01 ± 3.06	0.51
Prostate volume (mL)	51.65 (32.46, 81.68)	50.31 (38.73, 71.24)	0.96	54.05 (35.94, 70.01)	49.69 (37.35, 69.89)	0.67
Systolic pressure (mmHg)	132.00 (120.00, 142.00)	130.00 (120.00, 135.50)	0.21	130.00 (120.00, 140.00)	130.00 (120.00, 134.00)	0.54
Diastolic pressure (mmHg)	77.89 ± 11.23	77.79 ± 9.75	0.95	78.20 ± 11.22	77.75 ± 9.23	0.81
Fasting blood glucose (ng/mL)	5.11 (4.80, 5.60)	4.93 (4.40, 5.50)	0.05	5.06 (4.75, 5.57)	4.86 (4.40, 5.45)	0.09
Hypertension status (*n* [%])			0.38			0.21
Yes	12 (10.81%)	6 (7.14%)		8 (12.31%)	4 (6.15%)	
No	99 (89.19%)	80 (92.86%)		57 (87.69%)	61 (93.85%)	
History of smoking (*n* [%])			0.34			0.51
Yes	28 (25.23%)	27 (31.40%)		18 (27.69%)	15 (23.08%)	
No	83 (74.77%)	59 (68.60%)		47 (72.31%)	50 (76.92%)	
History of drinking (*n* [%])			0.57			0.55
Yes	29 (26.13%)	25 (29.76%)		19 (29.23%)	16 (24.62%)	
No	82 (73.87%)	61 (70.24%)		46 (70.77%)	49 (75.38%)	

**Table 2:** Baseline characteristics of patients used haemocoagulase agkistrodon for injection or hemocoagulase bothrops atrox for injection before and after propensity score matching.

Baseline	Before propensity score matching			After propensity score matching		
	Haemocoagulase agkistrodon (*N* = 109)	Hemocoagulase Bothrops Atrox (*N* = 99)	*p*	Haemocoagulase agkistrodon (*N* = 71)	Hemocoagulase Bothrops Atrox (*N* = 71)	*p*
Age (years)	72.87 ± 7.31	72.81 ± 7.40	0.95	73.45 ± 7.64	73.13 ± 7.46	0.81
Body mass index (kg/m^2^)	23.36 (20.76, 25.35)	23.02 (20.86, 25.34)	0.63	23.47 ± 3.65	22.81 ± 3.27	0.26
Prostate volume (mL)	51.46 (32.46, 79.88)	57.38 (37.01, 76.99)	0.47	51.65 (32.46, 77.62)	58.07 (37.52, 76.66)	0.46
Systolic pressure (mmHg)	132.00 (120.00, 140.00)	130.00 (120.00, 143.00)	0.83	132.73 ± 18.83	130.83 ± 16.93	0.53
Diastolic pressure (mmHg)	78.00 (70.00, 85.00)	80.00 (74.00, 88.00)	0.06	78.00 (69.00, 85.00)	80.00 (73.00, 84.00)	0.38
Fasting blood glucose (ng/mL)	5.11 (4.82, 5.59)	5.14 (4.71, 6.04)	0.87	5.10 (4.75, 5.55)	5.05 (4.59, 5.56)	0.48
Hypertension status (*n* [%])			0.20			0.44
Yes	13 (11.93%)	18 (18.37%)		10 (14.08%)	7 (9.86%)	
No	96 (88.07%)	81 (81.63%)		61 (85.92%)	64 (90.14%)	
History of smoking (*n* [%])			0.23			0.47
Yes	29 (26.61%)	34 (34.34%)		21 (29.58%)	25 (35.21%)	
No	80 (73.39%)	65 (65.66%)		50 (70.42%)	46 (64.79%)	
History of drinking (*n* [%])			0.76			0.85
Yes	27 (24.77%)	22 (22.92%)		19 (26.76%)	20 (28.17%)	
No	82 (75.23%)	77 (77.08%)		52 (73.24%)	51 (71.83%)	

**Table 3:** Baseline characteristics of patients used haemocoagulase agkistrodon for injection or tranexamic acid before and after propensity score matching.

Baseline	Before propensity score matching			After propensity score matching		
	Haemocoagulase agkistrodon (*N* = 111)	Tranexamic acid (*N* = 49)	*p*	Haemocoagulase agkistrodon (*N* = 38)	Tranexamic acid (*N* = 38)	*p*
Age (years)	72.72 ± 7.34	72.82 ± 5.75	0.93	72.61 ± 6.97	72.11 ± 5.87	0.74
Body mass index (kg/m^2^)	23.38 (20.62, 25.53)	22.96 (21.40, 24.42)	0.46	23.24 (21.72, 26.61)	23.10 (21.11, 24.77)	0.39
Prostate volume (mL)	51.65 (32.46, 82.32)	43.60 (30.66, 71.24)	0.43	52.38 (34.68, 79.88)	44.61 (32.65, 68.43)	0.81
Systolic pressure (mmHg)	132.00 (121.00, 143.00)	133.00 (120.00, 140.00)	0.98	133.55 ± 15.77	130.92 ± 15.63	0.47
Diastolic pressure (mmHg)	79.00 (70.00, 85.00)	80.00 (70.00, 90.00)	0.40	79.50 ± 12.24	79.63 ± 11.16	0.96
Fasting blood glucose (ng/mL)	5.12 (4.80, 5.60)	5.17 (4.42, 5.60)	0.61	5.12 (4.83, 5.59)	5.07 (4.51, 5.50)	0.36
Hypertension status (*n* [%])			0.08			0.53
Yes	13 (11.71%)	11 (22.45%)		5 (13.16%)	7 (18.42%)	
No	98 (88.29%)	38 (77.55%)		33 (86.84%)	31 (81.58%)	
History of smoking (*n* [%])			0.75			0.60
Yes	28 (25.23%)	13 (27.66%)		9 (23.68%)	11 (28.95%)	
No	83 (74.77%)	36 (72.34%)		29 (67.32%)	27 (71.05%)	
History of drinking (*n* [%])			0.69			0.61
Yes	30 (27.03%)	11 (23.91%)		12 (31.58%)	10 (26.32%)	
No	81 (72.97%)	38 (76.09%)		26 (68.42%)	28 (73.68%)	

**Table 4:** Baseline characteristics of patients given haemocoagulase agkistrodon for injection or ethylenediamine diaceturate injection before and after propensity score matching.

Baseline	Before propensity score matching			After propensity score matching		
	Haemocoagulase agkistrodon (*N* = 113)	Ethylenediamine Diaceturate (*N* = 37)	*p*	Haemocoagulase agkistrodon (*N* = 29)	Ethylenediamine Diaceturate (*N* = 29)	*p*
Age (years)	72.73 ± 7.31	71.14 ± 7.28	0.25	71.59 ± 7.41	71.69 ± 6.97	0.96
Body mass index (kg/m^2^)	23.47 ± 3.83	22.51 ± 2.68	0.11	23.54 ± 3.85	22.36 ± 2.79	0.19
Prostate volume (mL)	51.65 (33.89, 81.68)	48.35 (39.77, 73.58)	0.73	57.29 (34.80, 74.40)	46.31 (39.30, 73.89)	0.65
Systolic pressure (mmHg)	132.00 (121.00, 142.00)	126.00 (116.00, 130.00)	0.04	133.00 (125.00, 140.00)	130.00 (116.00, 135.00)	0.08
Diastolic pressure (mmHg)	79.00 (70.00, 85.00)	80.00 (72.00, 86.00)	0.18	77.45 ± 9.50	80.93 ± 9.93	0.18
Fasting blood glucose (ng/mL)	5.12 (4.82, 5.60)	4.97 (4.69, 5.40)	0.17	5.06 (4.75, 5.50)	4.86 (4.40, 5.32)	0.22
Hypertension status (*n* [%])			1			1
Yes	13 (11.50%)	4 (10.81%)		3 (10.34%)	4 (13.79%)	
No	100 (88.50%)	33 (89.19%)		26 (89.66%)	25 (86.21%)	
History of smoking (*n* [%])			<0.001			1
Yes	29 (25.66%)	21 (56.76%)		16 (55.17%)	16 (55.17%)	
No	84 (74.34%)	16 (43.24%)		13 (44.83%)	13 (44.83%)	
History of drinking (*n* [%])			0.71			0.77
Yes	30 (26.55%)	11 (29.73%)		9 (31.03%)	8 (27.59%)	
No	83 (73.45%)	26 (70.27%)		20 (68.97%)	21 (72.41%)	

**Table 5:** Effects of haemocoagulase agkistrodon for injection, hemocoagulase for injection, or hemocoagulase bothrops atrox for injection on patients after transurethral bipolar plasmakinetic prostatectomy.

Outcomes	Haemocoagulase agkistrodon (*N* = 65)	Hemocoagulase (*N* = 65)	*p*	Haemocoagulase agkistrodon (*N* = 71)	Hemocoagulase Bothrops Atrox (*N* = 71)	*p*
Hospitalization time (days)	7.00 (5.00, 8.00)	9.00 (8.00, 10.00)	<0.001	7.00 (6.00, 8.00)	8.00 (7.00, 10.00)	<0.001
Bladder irrigation time (hours)	41.00 (21.00, 64.00)	45.00 (23.00, 71.00)	0.06	45.00 (27.00, 71.00)	49.00 (45.00, 72.00)	0.04
Catheterization time (hours)	109.00 (88.00, 129.00)	164.00 (114.00, 189.00)	<0.001	114.00 (88.00, 143.00)	141.00 (120.00, 166.00)	<0.001
Urination unobstructed			0.68			0.36
Yes	63 (96.92%)	61 (93.85%)		70 (98.59%)	67 (94.37%)	
No	2 (3.08%)	4 (6.15%)				
Blood transfusion			1			1
Yes	1 (1.54%)	2 (3.08%)		1 (1.41%)	0 (0.00%)	
No	64 (98.46%)	63 (96.92%)		70 (98.59%)	75 (100%)	

**Table 6:** Effects of haemocoagulase agkistrodon for injection, tranexamic acid, or ethylenediamine diaceturate injection on patients after transurethral bipolar plasmakinetic prostatectomy.

Outcomes	Haemocoagulase agkistrodon (*N* = 38)	Tranexamic acid (*N* = 38)	*p*	Haemocoagulase agkistrodon (*N* = 29)	Ethylenediamine Diaceturate (*N* = 29)	*p*
Hospitalization time (days)	7.00 (6.00, 8.00)	7.00 (6.00, 9.00)	1	7.00 (6.00, 8.00)	10.00 (8.00, 11.00)	<0.001
Bladder irrigation time (hours)	44.00 (31.00, 80.00)	44.75 (39.00, 67.40)	0.99	46.00 (37.00, 71.00)	70.00 (45.00, 93.00)	0.10
Catheterization time (hours)	128.16 ± 55.94	123.57 ± 47.92	0.70	113.00 (95.00, 143.00)	160.00 (139.00, 168.00)	<0.001
Urination unobstructed			0.26			0.47
Yes	36 (94.74%)	32 (84.21%)		29 (100.00%)	27 (93.10%)	
No	2 (5.26%)	6 (15.79%)				
Blood transfusion			—			1
Yes	0 (0.00%)	0 (0.00%)		1 (3.45%)	0 (0.00%)	
No	38 (100%)	38 (100%)		28 (96.55%)	29 (100%)	

## Data Availability

The data used to support the findings of this study are included within the article and are available from the corresponding author upon request.
